# Injury of the optic radiation in patients with mild TBI: A DTT study

**DOI:** 10.1515/tnsci-2020-0108

**Published:** 2020-09-21

**Authors:** Sung Ho Jang, Seong Ho Kim, You Sung Seo

**Affiliations:** Department of Physical Medicine and Rehabilitation, College of Medicine, Yeungnam University, 317-1, Daemyungdong, Namku, Taegu, 705-717, Republic of Korea; Department of Neurosurgery, College of Medicine Yeungnam University, 317-1, Daemyungdong, Namku, Taegu, 705-717, Republic of Korea

**Keywords:** diffusion tensor imaging, diffusion tensor tractography, optic radiation, visual evoked potential, mild traumatic brain injury, head trauma

## Abstract

**Objectives:**

We investigated injuries of the optic radiations (ORs) in patients with mild traumatic brain injury (TBI) by using diffusion tensor tractography (DTT).

**Methods:**

Fifty-two consecutive patients who complained of visual problems showed abnormal visual evoked potential (VEP) latency but no abnormality on conventional brain MRI after mild TBI, and fifty normal control subjects were recruited for this study. Subjects’ ORs were reconstructed using DTT, and three DTT parameters (fractional anisotropy [FA], apparent diffusion coefficient [ADC], and tract volume) were measured for each OR.

**Results:**

Mean FA value and tract volume of the OR were significantly lower in the patient group than in the control group (*p* < 0.05). However, there was no significant difference in the ADC values of the OR between the patient and control groups (*p* > 0.05). A weak negative correlation was detected between VEP latency and OR fiber number (*r* = 0.204, *p* < 0.05).

**Conclusions:**

DTT revealed that OR injuries were not detected on the conventional brain MRI scans of patients who complained of visual problems and had abnormal VEP latency after mild TBI. Our results suggest that DTT would be a useful technique for detecting OR injury in patients with mild TBI.

## 1 Introduction

Traumatic brain injury (TBI) can be classified as mild, moderate, or severe based on assessment of the injury, and mild TBI comprises approximately 75% of all TBIs [1,2]. The visual system is vulnerable to TBI because several cranial nerves and about 30–40 cortical areas are involved in vision [1,2]. The prevalence of visual problems (e.g., oculomotor problems, visual field defects, visual information processing dysfunction, and visual attention deficits) in patients with TBI is high, approximately 50% of cases [3,4,5,6]. However, research on visual problems in mild TBI is rare; to the best of our knowledge, only one study has reported on the prevalence of visual problems in mild TBI. In that study, about 15% of mile TBI patients had visual problems (light sensitivity, 7%; blurred vision, 6%; double vision, 2%) [7]. Since the introduction of diffusion tensor imaging (DTI), several studies have described neural tract injuries in patients with mild TBI [8,9,10]. The demonstration of injury of neural tracts in patients with mild TBI is clinically important because such patients usually show no abnormality on conventional brain MRI [8,10,11,12,13]. Injury of the neural tracts after mild TBI has been demonstrated in the corticospinal tract, as well as in the fornix and cingulum [8,10,11,12,13]. However, little has been reported on mild TBI and the neural tracts involved in visual function, such as the optic radiation (OR) [11].

The OR is not easily distinguishable from adjacent neural structures. Therefore, a precise diagnosis of an OR injury is difficult when using conventional MRI or positron emission tomography [14,15,16]. However, diffusion tensor tractography (DTT), derived from DTI, allows three-dimensional reconstruction and evaluation of neural tracts, including the OR [14,16]. Although many studies have used DTI or DTT to describe OR injuries in patients with various brain pathologies including TBI [17,18,19], little has been reported about such injuries in mild TBI [9,20].

In this study, we used DTT to investigate OR injuries in patients with mild TBI.

## 2 Subjects and methods

### 2.1 Subjects

Fifty-two patients (20 males, 32 females; mean age: 45.9 ± 15.2 years, range: 18–72 years) with TBI who complained of visual problems and visited the rehabilitation department of a university hospital and 50 normal control subjects (23 males and 27 females; mean age: 42.2 ± 15.6 years, range: 21–75 years) were recruited for this study. The patients were recruited according to the following inclusion criteria: (1) loss of consciousness for less than 30 min, initial Glasgow Coma Scale score of 13–15, and posttraumatic amnesia for less than 24 h [1,21]; (2) no brain lesion detected on conventional MRI (*T*1-weighted, *T*2-weighted, fluid-attenuated inversion recovery, and *T*2-weighted gradient recall echo images); (3) more than 1 month after TBI onset; (4) age ranging from 18 to 75 years; (5) delayed visual evoked potential (VEP) latency; (6) complaints related to visual problems (e.g., visual defect, poor vision, or blurred vision); and (7) no history of head trauma or neurologic or psychiatric disease. No significant differences in age or sex compositions were detected between the patient and normal control groups (*p* > 0.05).

The VEP latent period was used to evaluate the status of the visual pathway. The normal VEP latency period reference values, by age and gender, were as follows: <107 ms (20–59 years for females), <110 ms (20–49 years for males, <115 ms (10–19 years for both sexes), <110 ms (60–69 years for females), and <120 m/s (50–69 years for males) [22].


**Informed consent:** Informed consent has been obtained from all individuals included in this study.
**Ethical approval:** The research has been complied with all the relevant national regulations, institutional policies, and in accordance the tenets of the Helsinki Declaration. The data were collected retrospectively, and the study protocol was approved by the appropriate institutional review board.

### 2.2 DTI

DTI data were acquired at an average of 5.2 ± 3.4 months after onset using a six-channel head coil on a 1.5 T Philips Gyroscan Intera MRI scanner. Imaging parameters were as follows: acquisition matrix = 96 × 96; reconstructed to matrix = 192 × 192 matrix; field of view = 240 mm × 240 mm; TR = 10,398 ms; TE = 72 ms; EPI factor = 5.9; *b* = 1,000 s/mm^2^; NEX = 1; slice gap = 0 mm; slice thickness = 2.5 mm.

**Figure 1:** (a) *T*_2_-weighted MR images show no abnormal lesion. (b) DTT for the injured OR (red arrow) and the VEP (latency: 151 m/s) of a patient (31-year-old male). (c) DTT of the OR and the VEP (latency: 100 m/s) of a normal subject (32 year old male).

Eddy current-induced image distortions were removed by using affine multiscale two-dimensional registration as provided in the Oxford Centre for Functional Magnetic Resonance Imaging of Brain Software Library (FSL; www.fmrib.ox.ac.uk/fsl) [23]. DTI-Studio software (CMRM, Johns Hopkins Medical Institute, Baltimore, MD, USA) was used for OR evaluation [24]. Fiber tracking was based on the fiber assignment continuous tracking algorithm and the multiple regions of interest (ROI) approach. To delineate the OR, a seed ROI was placed on the lateral geniculate body (LGB) on the color map, whereas the target ROI was placed on the color map at the OR bundle located in the middle portion between the LGB and the occipital pole [14,15]. Fiber tracking was performed based on a fractional anisotropy (FA) threshold of >0.15 and a direction threshold of <70° (Figure 1). We determined the FA, apparent diffusion coefficient (ADC), and tract volume of the OR in both hemispheres of each subject. DTI parameter values that were more than one standard deviation above or below the normal control values were defined as abnormal.

#### 2.2.1 VEPs

VEP measurements were obtained by using a Nicolet 1 channel LED goggle system. All procedures were performed with the subject in an awake state. The recording electrode was placed over the occipital cortex, and the amplitude and latency of the waveform generated were measured. Baseline flash goggle VEPs were recorded at O1/Cz (left visual cortex-to-vertex), Oz/Cz (midline visual cortex-to-vertex), and O2/Cz (right visual cortex-to-vertex) with OS (both eyes), OU (the right eye), and OD (the left eye) stimulation.

### 2.3 Statistical analysis

DTT data were analyzed by performing group-based analyses of the DTT parameters of the ORs in the patient and control groups. SPSS software (v. 15.0; SPSS, Inc., IBM Company, Chicago, Illinois, USA) was used for data analysis. The chi-squared test was used to examine the difference in sex compositions of the patient and control groups, and an independent *t*-test was used to assess age differences between the patient and control groups. Paired *t*-tests were used to assess the differences in DTT parameter values of the ORs of the patient and control groups. Pearson correlation coefficients were calculated to quantify the correlation between DTT parameters of the OR and clinical data (i.e., VEP latency). Null hypotheses of no difference were rejected if *p*-values were less than 0.05. A correlation coefficient of more than 0.60 indicated a strong correlation, a correlation coefficient between 0.40 and 0.59 indicated a moderate correlation, a correlation coefficient between 0.20 and 0.39 indicated a weak correlation, and a correlation coefficient less than 0.19 indicated a very weak relationship [25].

## 3 Results

A summary of the comparisons of the DTT parameters of the patient and control groups is presented in Table 1. The mean FA value and average tract volume of the ORs of the patient group were significantly lower than those in the control group (*p* < 0.05). However, no significant difference was detected between the ADC values of the ORs of the patient and control groups (*p* > 0.05) (Table 2).

**Table 1:** Visual problems of individual patients

No.	Age	Sex	Visual defect	Poor vision	Blurred vision
1	45	F	○	○	
2	23	F			○
3	56	F	○		
4	52	F		○	○
5	13	F	○	○	
6	50	F	○	○	
7	60	F		○	○
8	40	F		○	
9	35	F	○	○	
10	22	F	○	○	
11	56	F	○	○	
12	72	F		○	
13	65	F	○	○	
14	53	M	○	○	
15	42	M	○	○	
16	18	M	○	○	○
17	62	F	○	○	○
18	30	M	○	○	
19	46	M	○	○	
20	50	F	○	○	
21	49	F	○	○	
22	61	F	○		
23	56	F	○	○	
24	58	F	○	○	
25	33	F		○	
26	39	M	○	○	○
27	41	M	○	○	
28	56	M	○	○	
29	58	M	○	○	
30	63	F	○	○	
31	35	F	○	○	
32	65	F	○	○	
33	38	F	○	○	
34	38	M		○	
35	19	M		○	
36	25	F		○	
37	35	F		○	
38	59	F	○	○	
39	21	M	○	○	
40	31	M		○	
41	58	M	○	○	
42	58	F	○	○	
43	26	M		○	
44	63	F	○	○	
45	59	F	○	○	
46	61	F		○	
47	58	M		○	○
48	27	M	○	○	
49	21	M	○	○	
50	29	F	○	○	○
51	62	M		○	
52	65	M		○	

**Table 2:** Comparison of DTT parameters between the patient and control groups

	Patient group	Control group	*p*-Value
FA	0.47 (±0.11)	0.50 (±0.05)	0.042^a^
ADC	0.64 (±0.18)	0.60 (±0.04)	0.602
Fiber number	544.55 (±347.44)	1253.25 (±306.20)	0.001*

FA: fractional anisotropy, ADC: apparent diffusion coefficient, values represent patients: mean ± standard deviation (controls: mean ± standard deviation).

^a^Significant difference between the patient and control groups, *p* < 0.05.

A weak negative correlation was observed between the VEP latency values and fiber numbers of the ORs of the patient group (*r* = 0.204, *p* < 0.05) (Table 3).

**Table 3:** Correlation between DTT parameters and VEP latency

	FA	ADC	Fiber number
VEP latency	0.005	0.026	−0.214^a^

FA: fractional anisotropy, ADC: apparent diffusion coefficient, VEP: visual evoked potential.

^a^Significant difference between DTT parameter and VEP latency, *p* < 0.05.

## 4 Discussion

In this study, we investigated injury to the ORs in patients with visual problems and abnormal VEP latencies after the onset of mild TBI and determined the following: (1) FA and tract volume values of the ORs were significantly lower in the patient group than in the control group; (2) tract volume of the OR in the patient group was weakly negatively correlated with the VEP latency period.

The FA value represents the degree of directionality of microstructures, while the ADC value represents the magnitude of water diffusion [26,27,28]. Tract volume represents the number of voxels in a neural tract and is considered to indicate the number of fibers in that tract; therefore, a decrease in the fiber number indicates injury to a neural tract [29]. Decrements in FA and fiber number without a similar decrement in ADC in the patient group appears to indicate the presence of OR injuries in the patient group. Because the conventional brain MRI scans of the subjects in the patient group were normal, we suggest that the injury of these neural tracts was the result of traumatic axonal injury [30,31]. Furthermore, the weak negative correlation between VEP latency and OR fiber number suggests that a change in VEP latency reflects a change in the severity of an OR injury.

Since the introduction of DTI, many studies have used that imaging approach to document OR injury in patients with TBI [9,11,20,30,31,32,33,34,35]. The majority of these studies demonstrated the presence of OR injuries in patients with moderate or severe TBI [11,30,31,32,33,34,35]. Only a few similar studies of mild TBI have been reported [9,20]. In 2015, Jang and Seo investigated two patients with visual field defects in whom OR injuries were revealed on DTT [9]. During the same year, Vigneswaran et al. reported the decrements of FA values and increments of ADC values on DTI of the ORs in 61 patients with mild TBI compared with 19 normal control subjects [20]. To the best of our knowledge, this study is the first DTT-based study on patients with visual problems and abnormal VEP latencies after the onset of mild TBI. However, some limitations of this study should be considered. First, the fiber tracking technique is operator dependent. Second, DTT can produce false-negative results throughout the white matter of the brain due to fiber crossing or the partial volume effect [36,37]. Third, we could not investigate the relationship between the severity of visual problems and the magnitude of the DTT parameters because the clinical records presented presence or absence information, not severity-related information. Therefore, further prospective studies including detailed data related to visual problems should be encouraged.

In conclusion, by using DTT, we investigated OR injuries in patients who complained of visual problems and had VEP latency abnormalities after the onset of mild TBI. Our analysis of DTT parameters revealed the presence of OR injuries that were not detected on conventional brain MRI scans. Our results suggest that DTT would be a useful technique for detecting OR injuries in patients with mild TBI.
